# *Sigesbeckia orientalis* Extract Ameliorates the Experimental Diabetic Nephropathy by Downregulating the Inflammatory and Oxidative Stress Signaling Pathways

**DOI:** 10.1155/2022/3323745

**Published:** 2022-08-05

**Authors:** Chung-Ming Chen, Jer-Yiing Houng, Tsui-Ling Ko, Shu-Hui Juan, Hsiu-Chu Chou

**Affiliations:** ^1^Department of Pediatrics, School of Medicine, College of Medicine, Taipei Medical University, Taipei 11031, Taiwan; ^2^Department of Pediatrics, Taipei Medical University Hospital, Taipei 11031, Taiwan; ^3^Graduate Institute of Biotechnology and Chemical Engineering, I-Shou University, Kaohsiung 84001, Taiwan; ^4^Department of Nutrition, I-Shou University, Kaohsiung 82445, Taiwan; ^5^College of Science, National Sun Yat-Sen University, Kaohsiung 82445, Taiwan; ^6^Graduate Institute of Medical Sciences and Taipei Medical University, Taipei 11031, Taiwan; ^7^Department of Physiology, School of Medicine, College of Medicine, Taipei Medical University, Taipei 11031, Taiwan; ^8^Department of Anatomy and Cell Biology, School of Medicine, College of Medicine, Taipei Medical University, Taipei 11031, Taiwan

## Abstract

Diabetes in children and its complications are on the rise globally, which is accompanied by increasing in diabetes-related complications. Oxidative stress and inflammation induced by elevated blood sugar in diabetic patients are considered risk factors associated with the development of diabetes complications, including chronic kidney disease and its later development to end-stage renal disease. Microvascular changes within the kidneys of DM patients often lead to chronic kidney disease, which aggravates the illness. *Sigesbeckia orientalis* extract (SOE), reported to have strong antioxidative and excellent anti-inflammatory activities, is used in the modern practice of traditional Chinese medicine. Kidneys from three groups of control mice (CTR), mice with streptozotocin (STZ)-induced diabetes (DM), and mice with STZ-induced DM treated with SOE (DMRx) were excised for morphological analyses and immunohistochemical assessments. Only mice in the DM group exhibited significantly lower body weight, but higher blood sugar was present. The results revealed more obvious renal injury in the DM group than in the other groups, which appeared as greater glomerular damage and tubular injury, sores, and plenty of connective tissues within the mesangium. Not only did the DM group have a higher level of cytokine, tumor necrosis factor, and the oxidative stress marker, 8-hydroxyguanosine expression, but also factors of the nuclear factor pathway and biomarkers of microvascular status had changed. Disturbances to the kidneys in DMRx mice were attenuated compared to the DM group. We concluded that SOE is an effective medicine, with antioxidative and anti-inflammatory abilities, to protect against or attenuate diabetic nephropathy from inflammatory disturbances by oxidative stress and to cure vessel damage in a hyperglycemic situation.

## 1. Introduction

Diabetes mellitus (DM) is a metabolic disease characterized by hyperglycemia, caused by insulin deficiency (type I) or decreased insulin sensitivity (type II) [1]. Diabetes with onset from 6 months to early adulthood is classified as type I diabetes and is characterized by immune-mediated destruction of pancreatic beta cells, resulting in absolute insulin-deficient diabetes [2]. Exogenous insulin is the only treatment for patients to control hyperglycemia and control disease, so it is also known as insulin-dependent diabetes mellitus (IDDM) in the first worldwide accepted classification of diabetes [3]. Endothelial dysfunction caused by hyperglycemia, including a series of diabetic vasculopathy and related complications, has serious implications for the financial situation of individuals and their families, as well as the national economy [4, 5]. Complications of diabetic vasculopathy can include microvessels (eyes, kidneys, and nerves) and large vessels (heart and brain) [6, 7], which are major causes of high morbidity and mortality. The most common long-term complication in DM patients is nephropathy [8], which is the leading cause of the need for renal replacement therapy worldwide [9]. The main cause of diabetic nephropathy is hyperglycemia, which can eventually lead to end-stage renal disease (ESRD) requiring kidney transplantation, but most patients die of cardiovascular disease and infection before progressing to ESRD [10]. It was reported [11] that renal function decline was more pronounced in individuals with childhood/adolescent-onset type I diabetes.

Pathological renal microvascular changes in diabetic patients often contribute to chronic kidney disease and worsen diabetic status [12]. Hyperglycemia can cause metabolic changes and damage the kidneys, possibly due to a variety of cellular processes, including the production of advanced glycation end products, activation of the polyol pathway, activation of abnormal protein kinases, increased oxidative stress, and the encoding of certain molecules that regulate these genes involved in inflammation and extracellular matrix synthesis [13, 14]. The direct effect of hyperglycemia on the kidneys is to enhance the filtration and reabsorption of glucose to achieve the maximum function of the kidneys, resulting in increased glomerular filtration and increased tubular workload [15]. And then, glomerular endothelial dysfunction, glomerular basement membrane alterations, mesangial cell expansion, podocyte damage, and even sterile inflammation occur [16]. Hyperglycemia leads to endothelial dysfunction in vascular matrix synthesis and degradation, angiogenesis, and vascular permeability via interference with endothelial nitric oxide (NO) synthase (NOS; eNOS) activity and NO synthesis [17]. In our previous study, diabetic kidneys exhibited increased oxidative stress, inflammatory markers, and profibrotic growth factor in animals with experimental streptozotocin (STZ)-induced hyperglycemia [18].

Plants of the genus *Sigesbeckia* herbs are annual herbs widely distributed in tropical, subtropical, and temperate regions of the world. According to the species concept, there are about three to six species of *Sigesbeckia*, and one of the species, *S. orientalis* L., is a common weed in fallow fields of Taiwan [19]. Extracts from the whole plant of *Sigesbeckia* were reported to have strong antioxidative activity [20, 21] and anti-inflammatory and antirheumatism effects [22, 23]. Nuclear factor (NF)-*κ*B and mitogen-activated protein kinase (MAPK)-mediated reduction of inducible (i)NOS and cytochrome oxidase subunit 2 (COX2) are suggested to be involved in anti-inflammatory processes in *Sigesbeckia* plants [23]. The previous study evaluated 2,2-diphenyl-1-picrylhydrazyl (DPPH) radical scavenging activity, 2,2′-azino-bis (3-ethylbenzothiazoline)-6-sulphonic acid (ABTS) radical cation scavenging capacity, and reducing power to prove the antioxidant effects of *Sigesbeckia orientalis* extract on key enzymes associated with type 2 diabetes linked-*α*-amylase and *α*-glucosidase [24]. However, to the best of our knowledge, the effect of *Sigesbeckia orientalis* extract (SOE) on diabetes-induced hyperglycemia and its associated nephrotic complications has not been reported in the literature. Previous studies have demonstrated that hyperglycemia induces oxidative stress and inflammation in streptozotocin-induced diabetic kidneys. The current experiment tries to explore whether the effects of SOE will work on diabetic nephropathy and clarify its probable mechanisms.

## 2. Materials and Methods

### 2.1. Preparation of the SOE

Aerial parts of *S. orientalis* were purchased from Yuanshan Company (Kaohsiung City, Taiwan). The sample was identified, and its DNA polymorphism was reported [25]. The dried aerial part of *S. orientalis* was ground into a powder (9.3 kg) and extracted with 95% ethanol (47 L) for 1 day, and this process was repeated three times. After being filtered, a rotary evaporator was used to remove the solvent and concentrate the extracted solutions. The residue was then dried in a freeze-dryer, from which 489 g of dry mass was obtained. The chemical composition of the SOE was previously reported [26, 27].

### 2.2. Animals

This study was approved by the Institutional Animal Care and Use Committee of Taipei Medical University (license no. LAC-2016-0295) and according to protocols approved by the Association for the Evaluation and Accreditation of Laboratory Animal Care. BALB/cByJNarl male mice aged 4 weeks were purchased from the National Laboratory Animal Center (Taipei, Taiwan) a week before the experiments began. Animals were housed in metal cages with hardwood chip bedding with a 12 h light-dark cycle and free access to laboratory food with a standard chow diet (Rodent Laboratory Chow no. 5001, Ralston Purina Company, St. Louis, MO, USA) and water. The facility temperature was maintained at 20–23°C and the relative humidity was between 36 and 57%; at the same time, minimal environmental stress and basic environmental enrichment were carried out in strict accordance with the recommendations of our institutional guidelines. Blood sugar levels of all mice were measured with a One Touch II blood glucose meter (Lifescan, Milpitas, CA, USA) before beginning the experiments. At 6 h after the last feeding, the fasting blood sugar level was obtained from the tail vein of each animal. Blood sugar levels of the mice ranged from 110 ∼ 140 mg/dl.

### 2.3. DM Induced by STZ

Diabetes was induced by a single intraperitoneal injection of STZ dissolved in citrate buffer solution (0.01 M, pH 4.5) at a dose of 75 mg/kg body weight (BW) for 3 consecutive days. Control mice were treated with buffer only. At 48 h after the final injection, a blood sugar concentration of >270 mg/dl indicated a diabetic mouse. Prior to being sacrificed, the BW and blood glucose level of the mice were measured to confirm the persistence of DM.

### 2.4. Groups

Mice were assigned to either an STZ-induced diabetes with hyperglycemia (with a fasting blood sugar level of >270 mg/dl) (DM) group or a control (CTR) group. Mice in the DM group were randomly subdivided into DM mice with no treatment as the DM subgroup and DM mice were treated daily with 88 mg/kg of SOE by oral gavage for 8 weeks as the DMRx subgroup. Further experiments continued following the treatment period.

### 2.5. Tissue Preparation

At the end of the treatment period, all mice were sacrificed. The animals were intramuscularly anesthetized using a combination of ketamine (8 mg/100 g·BW), xylazine (2 mg/100 g·BW), and atropine (0.16 mg/100 g·BW). The left kidney was removed and fixed in 4% paraformaldehyde for 48 h, washed in phosphate-buffered saline (PBS), and serially dehydrated in increasing concentrations of ethanol before being embedded in paraffin for histologic assessment and immunohistochemical processing.

### 2.6. Histological Assessment and Morphological Analysis

Hematoxylin and eosin (H&E), periodic acid Schiff (PAS), and Masson's trichrome staining were performed after routine deparaffinization of serial 5-micron-thick paraffin tissue sections, followed by light microscopy to assess the kidney morphology. Histological analysis of renal tubular injury was assessed with a modification of the method of Kurus et al. [28]; tubular injury was defined as tubular dilation, tubular atrophy, vacuolization, tubular epithelial cell degeneration and shedding, and thickening tubular basement membrane. The degree of tubular injury was evaluated according to the following scoring system: 0, no tubular injury; 1, ≤10% of tubules injured; 2, 10% ∼ 25% of tubules injured; 3, 26% ∼ 50% of tubules injured; 4, 51% ∼ 75% of tubules injured; and 5, ≥75% of tubules injured. Histological analyses of the proportion of glomeruli in the cortex and the size of individual glomeruli were performed according to a modification of the method of Toledo-Rodriguez et al. [29]. The sizes of individual glomeruli located in the intermediate cortex and juxtamedullary zone were calculated as the average of the largest and smallest glomerular diameters in the field of view; the calculations included 10 ± 5 glomeruli per kidney. To assess the extent of glomerular damage, PAS-stained sections were examined using a semiquantitative scoring system, which was modified from the system used in the study by Raij et al. [30]. The mean optical density values of 10 nonoverlapping microscopic fields of Masson's trichrome-stained kidney sections from each animal were analyzed using Image-Pro Plus 6.0 (Media Cybernetics, Bethesda, MD, USA) to assess the presence of collagen [31].

### 2.7. Immunohistochemistry

Heat-induced epitope retrieval was performed by immersing the slides in 0.01 M sodium citrate buffer (pH 6.0) after routine deparaffinization, to block endogenous peroxidase activity and nonspecific antibody binding, the antigen-retrieved sections were then preincubated in 0.1 M·PBS containing 10% normal goat serum and 0.3% H_2_O_2_ for 1 h at room temperature. After previous process, sections were incubated with rabbit polyclonal anti-tumor necrosis factor (TNF)-*α* (1 : 100; Gene Tax, Irvine, CA, USA), anti-nuclear factor-*κ*B p65 (NF-*κ*B), anti-Von Willebrand factor (VWF) (1 : 100; Abcam, Cambridge, MA, USA), and mouse monoclonal anti-8-hydroxy-2′-deoxyguanosine (8-OHdG) (1 : 100; Abcam), anti-nitric oxide (NO) synthase 3 (NOS3 (A-9)), anti-NF-kappa-B inhibitor alpha (I*κ*B*α* (H-4)), and anti-I*κ*B kinase inhibitor (IKK-i (A-11)) (1 : 50; Santa Cruz Biotechnology, Santa Cruz, CA, USA) antibodies as primary antibodies for 20 h at 4°C. Sections were subsequently treated for 1 h at 37°C with biotinylated goat anti-rabbit immunoglobulin G (IgG; 1 : 200, Vector Laboratories, Burlingame, CA, USA) for the anti-TNF-*α*, anti-NF-*κ*B, and anti-VWF antibodies and with biotinylated goat anti-mouse IgG (1 : 200; Jackson ImmunoResearch Laboratories, West Grove, PA, USA) for the anti-8-OHdG, anti-NOS3, anti-I*κ*B*α*, and anti-IKK-i antibodies. Then, sections were reacted with reagents from an avidin-biotin complex kit (Vector Laboratories), and brown reaction products were visualized using a diaminobenzidine substrate kit (Vector Laboratories) according to the manufacturer's recommendations. All immunostained sections were examined and photographed with a Nikon Eclipse E600 Microscope (Nikon, Tokyo, Japan). At 400× magnification, five randomly selected fields from each section at 400× magnification were photographed using a digital camera and imported into a computerized image analysis system (Image-Pro Plus 6.0 for Windows, Media Cybernetics, Silver Spring, MD, USA). Immunoreactive positive 8-OHdG and NF-*κ*B nuclei were quantified using an automated object counting and measurement process, yielding a percentage of positively stained cells; these values were expressed as a labeling index (%) for 8-OHdG and NF-*κ*B [32]. Mean optical density values of TNF-*α*-, IKB*α*-, and IKK-I-positive staining in five randomly selected fields from each section were obtained. The mean eNOS-(NOS3) and VWF-stained vessel densities were counted in an unbiased manner, and at least five random lung fields at 400× magnification were counted as modified by Irwin et al. [33].

### 2.8. Statistical Analysis

All data are expressed as the mean ± standard deviation (SD). The *P* values for difference in means between the two conditions was calculated using the unpaired Student's *t*-test, and difference among between groups was tested using analysis of variance (ANOVA) (one-way ANOVA, Fisher's test). Differences were considered statistically significant at *P* < 0.05.

## 3. Results

### 3.1. Effect of SOE on BW Gain and Blood Glucose Levels in Mice with STZ-Induced Diabetes

Mean body weight and blood glucose levels prior to the start of the experiment were comparable between the CTR, DM, and DMRx groups (for BW: CTR = 21.8 ± 2.4 g, DM = 22.3 ± 1.6 g, and DMRx = 22.8 ± 0.5 g; for blood glucose: CTR = 126.0 ± 5.2 mg/dl, DM = 127.3 ± 5.3 mg/dl, and DMRx = 129.1 ± 7.2 mg/dl) (Table 1). Within 2 days after STZ injection, the blood glucose level of the diabetic-induced animals increased to 270 ∼ 500 mg/dl. At the end of the experimental period, mice with STZ-induced diabetes (DM) displayed lower BW gain (CTR = 25.2 ± 1.5 g, DM = 22.6 ± 0.5 g, and DMRx = 23.3 ± 1.0 g, *P* < 0.01) and a significantly higher fasting plasma glucose level than did control mice (CTR) and diabetic mice daily treated with the SOE (DMRx) for 8 weeks (CTR = 120.3 ± 5.5 mg/dl, DM = 373.9 ± 19.8 mg/dl, and DMRx = 286.5 ± 34.0 mg/dl, *P* < 0.01). In subjects with SOE supplementation, mean BW and blood glucose levels significantly differed from the DM group (*P* < 0.05). The SOE could partially alleviate the hyperglycemia induced by STZ.

### 3.2. Hyperglycemia Is Highly Associated with Renal Damage, Which SOE Can Mitigate

The morphology of kidney tissues was disturbed by STZ-induced DM, which was evident in glomeruli, renal tubules, and blood vessels. Dilated renal tubules were filled with an eosinophilic colloid substance in the lumen instead of at the intact brush border, and tubular cells were condensed and detached from the wall, as shown in Figure 1(a). The lumen of the glomerular capillaries of the control was less dilated than those in the DM and DMRx groups. The diabetic kidney exhibited a significantly lower proportion of the cortex occupied by glomeruli but higher tubular injury scores and a greater glomerular profile size than did control and SOE-treated mice (Figure 1(b); *P* < 0.01). PAS stain is usually used to estimate the structural damage of renal tubules and glomeruli. The mesangium was more expansive between the capillaries, and the basement membrane of glomerular capillaries was thicker in DM kidneys than in the CTR and DMRx groups (Figure 2(a)), which was clearly evident by the higher glomerular injury score in mice with STZ-induced DM according to the morphometric analysis (Figure 2(c); *P* < 0.01). In diabetic kidneys, the brush border was disturbed in the proximal convoluted tubules and the enlarged lumen had lost its cellular integrity and had shed its lining as observed in convoluted renal tubules. Formerly described situations were occasionally present in kidneys from the control and SOE-treated groups. Masson's trichrome is a stain commonly used to assess collagen fiber deposition and to verify the presence of renal fibrosis. Interstitial spaces of kidney tissues from hyperglycemic mice were conspicuously stained with Masson's trichrome (Figure 2(b)). Kidney tissues of CTR and DMRx mice were significantly less stained with Masson's trichrome than was the DM group (Figure 2(d)). Both the glomerular damage score and Masson's trichrome optical density in the interstitial spaces of the kidney were reduced by SOE supplementation (*P* < 0.01).

### 3.3. The SOE Restores the Histochemical Characters of the Microvascular in Kidneys from Hyperglycemic Mice

Vessels in the kidneys were examined at the glomeruli and interstitial spaces between the renal tubules of the cortex and medulla. IHC reactivities of VWF as in Figure 3(a) and eNOS as in Figure 3(b) in kidney sections were mainly present in endothelial cells of the glomeruli and vessels of the renal cortex and medulla. Expression patterns of VWF and eNOS in endothelial cells of the kidney had changed in diabetic animals. The expression tendency of VWF was opposite to that of eNOS, with eNOS, but not VWF, immunostaining endothelial cells, which displayed greater numbers in the CTR and DMRx groups than the DM group (see Figures 3(c) and 3(d)). Results of the morphometric analysis reflected higher VWF- and lower eNOS-positive vascular densities in diabetic kidneys than in the CTR or DMRx groups (*P* < 0.01). After having received the SOE, VWF- and eNOS-immunostained vessels were restored in the kidneys of diabetic mice to an extent that they were comparable to the control group.

### 3.4. The SOE Arrests Oxidative Stress Induced by Hyperglycemia

There was less 8-OHdG immunoreactivity observed in the cells of kidneys of the control and SOE-treated DM mice; see Figure 4(a). The oxidative stress marker, 8-OHdG, existed in the nuclei of podocytes, endothelial cells, and tubular cells. Kidneys with STZ-induced diabetes with no treatment displayed increased 8-OHdG-positive cells in both the cortex and medulla. Quantitative analysis of 8-OHdG-positive cells was performed in kidneys from each group (Figure 4(b)), and the results showed more reacted cells in kidneys with STZ-induced diabetes than in the other groups (*P* < 0.01).

### 3.5. Regulators of the NF-*κ*B Signaling Pathway and TNF-*α* Expression in Diabetic Kidney Are Precluded by the SOE

The current results indicated that IHC reactions of IKK-i (Figure 5(a)), I*κ*B*α* (Figure 5(b)), NF-*κ*B (Figure 5(c)), and TNF-*α* (Figure 6(a)) in kidney tissues changed after diabetes was induced. The immunoreactivity of IKK-i, NF-*κ*B, and TNF-*α* was predominantly present in the cytoplasm and was observed not only in tubular cells but also in endothelial cells and podocytes. NF-*κ*B-immunostained nuclei were found in podocytes, endothelial cells, and tubular cells. Except for I*κ*B*α*, IKK-i−, NF-*κ*B−, and TNF-*α*-immunostained cells were more prominently present in kidney sections of diabetic mice than in the control or SOE-supplemented groups. Evidence from the morphometric analysis showed that the optical densities of both IKK-i (Figure 5(d)) and TNF-*α* (Figure 6(b)) and the labeling density of NF-*κ*B (Figure 5(f)) were significantly higher in the DM group than the other groups (*P* < 0.01). In contrast to the results of IKK-i, NF-*κ*B, and TNF-*α*, the expression of I*κ*B*α* (Figure 5(e)) was reduced in diabetic kidney sections. In the kidneys of DM mice, SOE decreased the immunoreactivity of IKK-i, NF-*κ*B, and TNF-*α*, while it increased the expression of I*κ*B*α*.

## 4. Discussion

Histological and immunohistochemical examinations were designed in this study to compare kidney tissue from mice with experimentally induced hyperglycemia with those from mice administered SOE after induction of hyperglycemia. The results revealed that, in addition to increasing the immunoreactivity of 8-OHdG in the kidney tissue of STZ-induced diabetic mice, the expression levels of IKK-i, NF-*κ*B, and TNF-*α* were significantly increased, but the immunoreactivity of IKK-i was decreased. Furthermore, renal vascular endothelial cells in STZ-induced diabetic mice showed attenuated eNOS but significant VWF immunostaining. SOE supplementation alleviated the parenchymal and microvascular status of kidney tissues induced by hyperglycemia.

A large number of chronic diseases are associated with the production of reactive oxygen species (ROS), which lead to oxidative stress and oxidation of various proteins [34], resulting in damage of cellular molecules such as DNA, proteins, and lipids [35]. It was demonstrated that hyperglycemia induces oxidative stress as exhibited by significantly higher expression of 8-OHdG, which activates inflammatory cytokines via NF-*κ*B signaling in diabetic kidneys and lungs [36, 37]. Almost all danger-sensing receptors of the immune system activate NF-*κ*B transcription factors to mediate effector functions. Lots of stimuli activate NF-*κ*B, primarily through IKK-dependent phosphorylation and subsequent degradation of I*κ*B proteins. Released NF-*κ*B dimers enter nucleus, where they regulate the transcription of multiple genes that encode cytokines, growth factors, cell adhesion molecules, and pro- and antiapoptotic proteins [38, 39]. I*κ*B*α* is a member of a family of cellular proteins that function as an inhibitor of NF-*κ*B transcription factor [40]. IKK phosphorylates inhibitors of NF-*κ*B and I*κ*B*α*, leading to dissociation of the I*κ*B*α*/NF-*κ*B complex and then degradation of the inhibitor. IKK was suggested to act as an I*κ*B kinase in the immune system [41].

Chronic inflammation and oxidative stress not only are key factors in the progression of hyperglycemia-induced diabetic nephropathy, but also serve as mediators of apoptotic signaling that trigger cellular and tissue damage leading to organ failure [42–44]. As demonstrated by Piconi et al. [45], when D-sugar acid 1,4-lactone (DSL), known for its detoxification and antioxidant properties, was administered to diabetic rats, renal function was improved by inhibiting oxidative stress-related signaling pathway. 8-OHdG is a DNA base-modified product generated by ROS and serves as a marker of oxidative DNA damage. Measuring the products of 8-OHdG by a quantitative IHC assay is a useful tool for estimating oxidative stress in an organism [46, 47]. In this study, we assessed histological changes, but analyses of 8-OHdG expression and factors related to the NF-*κ*B signaling pathway and the inflammatory cytokine, TNF-*α*, were used to detect the efficiency and possible mechanisms of SOE supplementation in the kidneys of hyperglycemic animals. It was observed that structures of the kidney were disturbed by hyperglycemia, but such disturbances were ameliorated by the SOE. Not only did the SOE decrease the immunoreactivity of the oxidative stress marker, 8-OHdG, but also the expression levels of nuclear NF-*κ*B and the cytokine, TNF-*α*, were dramatically reduced in diabetic kidneys. In kidney tissues from diabetic mice, the expression of the NF-*κ*B inhibitor, I*κ*B*α*, was decreased, but that of IKK, which dissociates the I*κ*B*α*/NF-*κ*B complex, was increased. All of these situations provide evidence to explain that diabetic renal tissues were suffering from oxidative stress and inflammation. As demonstrated by Noordin et al. [48], oral administration of an aqueous extract of the flowers of *Etlingera elatior*, a medicinal plant of the ginger family Zingiberaceae for 6 weeks, reduced blood sugar and inflammatory markers and enhanced antioxidant markers, thereby against diabetic nephropathy in rat. According to our experimental data, we believe that SOE rescued diabetic nephropathy through its antioxidant and anti-inflammatory abilities.

It was reported that oxidative stress is associated with diabetic vascular complications, which impair the vascular wall and cause endothelial dysfunction [17, 49] and are considered to play a considerable role in the pathogenesis of cardiovascular diseases, neuropathy, nephropathy, and retinopathy [50–52]. Microvascular changes within the kidneys of DM patients often lead to chronic kidney disease which aggravates the illness [12]. Hyperglycemic activation of the aldose reductase pathway changes the NADH/NAD^+^ ratio and results in increased production of oxidative stress. Endothelial cells suffering from the cytotoxic effects experience reduced availability of NO [53]. Insulin was demonstrated to induce eNOS expression in endothelial cells grown from the human aorta, but the inflammatory cytokine, TNF-*α*, had an inhibitory effect on insulin-induced eNOS expression [54, 55]. eNOS messenger (m)RNA expression levels in tissues of the kidneys, heart, aorta, and sciatic nerve from rats after 4 weeks of hyperglycemia were significantly downregulated. Antioxidative treatment reversed eNOS expression, which was proposed as a possible important therapeutic option for preventing vascular damage in DM [56]. Information from in vitro and in vivo studies indicated that oxidative stress and hyperglycemia downregulated the expression of eNOS, whereas insulin and antioxidative supplementation could induce eNOS expression. VWF was proposed and demonstrated to be a biomarker of vascular injury in cardiovascular diseases, such as diabetes, stroke, and coronary artery disease [57–59]. Different mediators of inflammation, such as cytokines and superoxide anions, produce an increase in VWF levels through various mechanisms [53, 59]. The VWF was significantly increased in insulin-requiring diabetes, which indicated diabetic endothelial injury and damage were the primary mechanisms contributing to an increased occurrence of vascular and cardiac events in diabetic postinfarction patients [60]. Distribution patterns of blood vessel-bound factors of VWF and eNOS in the current study were used to confirm that the status of vascular disturbances caused by hyperglycemia could be overcome with SOE treatment.

SOE treatment may cause potential side effects in animals, as discussed in several previous studies that have examined chronic toxic effects of body organs through long-term SOE treatment. Rats were treated with SOE for 24 weeks [61] or 6 months at a dose of 5 g/kg·BW/daily [62]. Following these treatments, rats had demonstrated reduced body weight gain, histopathological damage to the liver and lung, treatment-induced oxidative stress, inflammation, and MAPK activation. In the current study, the dose of SOE was daily administrated 88 mg/kg BW for 8 weeks, the dose of SOE was shown to be effective in DM, and the above events were not observed. It should be that we used significantly less doses and time duration than previous studies. As a precaution, these potential consequences should be addressed in future clinical applications.

## 5. Conclusions

The current study expounded that hyperglycemia-induced oxidative stress evokes inflammatory pathway development, and then elevated proinflammatory cytokines disturb vessels and promote nephropathic progression. SOE supplementation attenuated oxidative stress and inflammatory situations and affected the expression patterns of eNOS and VWF in the kidneys of diabetic mice and thus helped maintain the morphologic intactness of diabetic kidney tissues. This study provides the positive effects of traditional medicine- *Sigesbeckia orientalis,* downregulating the oxidative stress and inflammatory pathways of experimental diabetic kidney, may provide a remedy to improve the life quality of children and adolescents suffering diabetic nephropathy. The SOE-related issues are being further studied so that it can accurately provide the prevention and treatment of diabetic nephropathy and related complications.

## Figures and Tables

**Figure 1:** Representative photographs of H&E-stained kidney sections (a) and morphometric analysis of the proportion of the cortex occupied by glomeruli, the glomerular profile size, and tubular injury score (b) from control (CTR), diabetic mellitus (DM), and DM *Sigesbeckia orientalis* extract (SOE)-administrated (DMRx) mice. Kidney sections from animals in the CTR group revealed no significant histological changes. Extensive alterations after diabetes were induced by a streptozotocin (STZ) injection (DM). The eosinophilic colloid substance (white asterisk) present in dilated renal tubules (black asterisk) was observed in DM kidney sections. A renal tubule is displayed with severe disturbance as condensed tubular cells detached from the basement membrane (black arrow), attenuated brush borders, and caused loss of the intact morphology of the renal tubule. Except for the dilated renal tubules, none of the morphological changes that existed in the DM group was found in renal sections of the SOE group. The lumen of glomerular capillaries was more dilated in mice with DM than in CTR mice. Mice with DM without SOE treatment exhibited a decreased number of renal corpuscles, an enlarged glomerular profile, and an obviously higher injury score. Data are presented as the mean ± SD. ^*∗*^*P* < 0.01 vs. the CTR or DMRx group.

**Figure 2:** Representative photographs of periodic acid Schiff (PAS)-stained cortex (a) and Masson's trichrome-stained medulla (b) of kidney tissues from control (CTR), diabetes mellitus (DM), and DM with *Sigesbeckia orientalis* extract (SOE)-administrated (DMRx) mice. Semiquantitative analyses of glomerular damage scores and the degree of interstitial connective tissue deposition are, respectively, provided in (c) and (d). The mesangium had increased between the glomerular capillaries (white asterisk), and the basement membrane (white arrows) of the capillary was thickened in glomeruli of DM kidneys. Some detached tubular cells (black arrow) from the distal convoluted tubules in the diabetic kidney cortex were observed. Numerous PAS-stained brush borders (black asterisk) are displayed in the proximal convoluted tubules in the CTR and DMRx groups, but they were reduced in the DM group. Notable connective tissue between the renal tubules (black arrow) in the medulla was detected in kidneys of DM mice. Kidney tissues from diabetic mice showing significantly higher glomerular damage scores and increased optical density in connective tissues stained with Masson's trichrome. Data are presented as the mean ± SD. ^*∗*^*P* < 0.01 vs. the CTR or DMRx group.

**Figure 3:** Representative photographs of kidney sections from control (CTR), diabetes mellitus (DM), and DM with *Sigesbeckia orientalis* extract (SOE)-administered (DMRx) mice, which were immunoreacted with Von Willebrand factor (VWF) (a) and endothelial nitric oxide synthase (eNOS) (b). The VWF-(c) and eNOS-stained (d) vessel numbers per field are displayed simultaneously. The VWF-immunostained vascular density of kidneys in DM mice was higher, but the eNOS-immunostained density was lower than in the CTR and DMRx groups. Data are presented as the mean ± SD. ^*∗*^*P* < 0.01 vs. the CTR or DMRx group.

**Figure 4:** Representative photographs show 8-hydroxy-2′-guanosine (8-OHdG) IHC-stained kidney sections from control (CTR), diabetes mellitus (DM), and DM *Sigesbeckia orientalis* extract (SOE)-administered (DMRx) mice (a) and semiquantitative detection of the 8-OHdG-labeled nucleus number index in each group (b). Hyperglycemic (DM) mice had numerous 8-OHdG-labeled nuclei (black arrows), and the labeling index results demonstrated a significant difference between DM mice and the other groups. Data are presented as the mean ± SD. ^*∗*^*P* < 0.01 vs. the CTR or DMRx group.

**Figure 5:** Representative photographs of kidney sections of control (CTR), diabetes mellitus (DM), and DM with *Sigesbeckia orientalis* extract (SOE)-administered (DMRx) mice. All sections were immunoreacted for I*κ*B kinase inhibitor (IKK-i) (a), nuclear factor-*κ*B inhibitor alpha (I*κ*B*α*) (b), and nuclear factor (NF)-*κ*B (c). Positive immunostaining of IKK-i and I*κ*B*α* was obviously present in the cytoplasm in all groups, and kidney sections of the DM group predominantly reacted with IKK-i but mildly with I*κ*B*α*. The immunoreactivity of NF-*κ*B nuclei (black arrows) was numerous in mice with hyperglycemia (DM). Significant differences in IKK-I (d), I*κ*B*α* (e), and NF-*κ*B (f) immunostaining between the DM group and the other groups were demonstrated using a semiquantitative analysis. Data are presented as the mean ± SD. ^*∗*^*P* < 0.01 vs. the CTR or DMRx group.

**Figure 6:** Representative photographs of kidney sections from control (CTR), diabetes mellitus (DM), and DM with *Sigesbeckia orientalis* extract (SOE)-administered (DMRx) mice immunostained for tumor necrosis factor (TNF)-*α* (a) and a semiquantitative analysis (b) are provided concurrently. TNF-*α* (black arrows) protein expression was detected in nuclei and the cytoplasm of podocytes and tubular cells, and the immunoreactivity was more intense and extensive in diabetic kidneys than in CTR and DMRx mice. Data are presented as the mean ± SD. ^*∗*^*P* < 0.01 vs. the CTR or DMRx group.

**Table 1:** Body weights (BWs) and blood glucose (BS) levels before the experiment and after being sacrificed of control mice (CTR), mice with streptozotocin-induced diabetes (DM), and DM mice with the *Sigesbeckia orientalis* extract (SOE) administered at 88 mg/kg/daily by oral gavage for 8 weeks after diabetes was induced (DMRx).

Group	*n*	Initial BW (g)	Final BW (g)	Initial BS (mg\dl)	Final BS (mg\dl)
CTR	7	21.8 ± 2.4	25.2 ± 1.5	126.0 ± 5.2	120.3 ± 5.5
DM	6	22.3 ± 1.6	22.6 ± 0.5^*∗*^	127.3 ± 5.3	373.9 ± 9.8^*∗*^
DMRx	10	22.8 ± 0.5	23.3 ± 1.0^*∗*^^,#^	129.1 ± 7.2	286.5 ± 34.0^*∗*^^,#^

Data are presented as the mean ± SD. ^*∗*^Significantly different from the control (CTR) group, *P* < 0.01; and ^#^significantly different from the DM group, *P* < 0.05.

## Data Availability

The datasets used to support the findings of this study are available from the corresponding author upon request.
